The article "A Computational Model to Investigate GABA-Activated Astrocyte Modulation of Neuronal Excitation" was published in 2020. Journal: Comput Math Methods Med.

# A Computational Model to Investigate GABA-Activated Astrocyte Modulation of Neuronal Excitation

**DOI:** 10.1155/2020/8750167

**Published:** 2020-09-15

**Authors:** Licong Li, Jin Zhou, Hongji Sun, Jing Liu, Hongrui Wang, Xiuling Liu, Changyong Wang

**Affiliations:** ^1^College of Physics Science and Technology, Hebei University, Baoding 071002, China; ^2^Key Laboratory of Digital Medical Engineering of Hebei Province, Hebei University, Baoding 071002, China; ^3^Department of Neural Engineering and Biological Interdisciplinary Studies, Institute of Military Cognition and Brain Sciences, Academy of Military Medical Sciences, Beijing 100850, China; ^4^Brainnetome Center, Institute of Automation, Chinese Academy of Sciences, Beijing 100190, China

## Abstract

Gamma-aminobutyric acid (GABA) is critical for proper neural network function and can activate astrocytes to induce neuronal excitability; however, the mechanism by which astrocytes transform inhibitory signaling to excitatory enhancement remains unclear. Computational modeling can be a powerful tool to provide further understanding of how GABA-activated astrocytes modulate neuronal excitation. In the present study, we implemented a biophysical neuronal network model to investigate the effects of astrocytes on excitatory pre- and postsynaptic terminals following exposure to increasing concentrations of external GABA. The model completely describes the effects of GABA on astrocytes and excitatory presynaptic terminals within the framework of glutamatergic gliotransmission according to neurophysiological findings. Utilizing this model, our results show that astrocytes can rapidly respond to incoming GABA by inducing Ca^2+^ oscillations and subsequent gliotransmitter glutamate release. Elevation in GABA concentrations not only naturally decreases neuronal spikes but also enhances astrocytic glutamate release, which leads to an increase in astrocyte-mediated presynaptic release and postsynaptic slow inward currents. Neuronal excitation induced by GABA-activated astrocytes partly counteracts the inhibitory effect of GABA. Overall, the model helps to increase knowledge regarding the involvement of astrocytes in neuronal regulation using simulated bath perfusion of GABA, which may be useful for exploring the effects of GABA-type antiepileptic drugs.

## 1. Introduction

The brain is an adaptive nonlinear dynamic system, in which excitatory-inhibitory (EI) balance is vital for normal brain function [1]. Regulation of neuronal excitability is one of the key factors in achieving EI balance. Among the regulatory transmitters involved in neuronal excitability, GABA, released by the GABAergic neurons or astrocytes [2, 3], is the major inhibitory transmitter, which decreases neuronal excitability and prevents the neurons from overfiring. It is well established that GABA plays a central role in memory consolidation [4], motor coordination [5], and motor learning [6]. The dysregulation of GABA is closely related to certain neurological disorders, such as epilepsy [7, 8], Parkinson's disease [9], and anxiety and depression [10]. Experimental studies and the computational models have increased our understanding of the significant functions of GABA. Many reports suggest that elevated GABA concentrations exert both inhibitory and excitatory effects on neuronal firing [11–13]. Such contradictory scenario has also been reported in bath perfusion of a GABA_B_R agonist [14, 15]. One potential mechanism is that elevation in ambient GABA concentration can reduce the inhibitory effect of GABAergic synapses on the connected excitatory neurons, resulting in an overall increase in excitability via the disinhibition of the neurons [12, 14].

Due to the tight morphological arrangement of the astrocytes and neurons, named “tripartite synapses” [16], astrocytes actively participate in the modulation of neuronal activity and synaptic behavior (for reviews, see [17–19]). Recent studies have demonstrated that GABA-activated astrocytes in the hippocampus or cortex can induce depolarized current and enhance neuronal excitability via the release of gliotransmitter glutamate [20, 21]. These findings initiate a discussion regarding astrocytes as modulators in the conversion of inhibitory stimuli to excitatory signals, which provide novel insight into the function of astrocytes in terms of neural network excitation. However, the signaling machinery involved in the intracellular cascade of GABA_B_R-mediated Ca^2+^ increase and glutamate release in astrocytes remains unclear [20]. In this case, computation modeling can be used as a viable alternative to understand the role of GABA-activated astrocytes in the regulation of neuronal excitation. Most astrocyte models are based on the Ca^2+^ dynamics models [22, 23], which are overwhelmingly driven by synaptically released glutamate [24–26]. According to the existing glutamate-activated astrocyte mathematical framework, Li et al. developed a GABA-activated astrocyte model coupled to the seizure-firing neurons [27]. In particular, the astrocyte model added a complex differential equation and involved dual signaling of GABA released by interneuron and glutamate released by astrocyte. Nevertheless, an accurate description of the regulation of the excitatory neurons by GABA-activated astrocytes remains elusive.

In the present study, we addressed this issue by devising a novel neuron-astrocyte interaction computational model and simulating injection of exogenous GABA (“virtual” GABA, [GABA_ex_] = 0 *μ*M, 1 *μ*M, 5 *μ*M, and 10 *μ*M) into the extracellular space. The goal of this paper was to describe neuronal population activity and investigate the modulation of astrocytes on the neurons in stimulus conditions by lumping the microscale tripartite synapse model and macroscale neuronal-astrocytic network. On the cell level, the GABA-activated astrocyte model was incorporated into a modeling framework of glutamatergic gliotransmission [28]. The model described the activation of astrocytes by synaptic glutamate, in addition to the crosstalk between the GABA_B_Rs and mGluRs to induce astrocytic calcium elevation [29]. By considering these two signaling pathways, we may better understand the effect of GABA on astrocytes. Furthermore, synaptic regulation by astrocyte-derived glutamate is not a straightforward process in contrast to the previous synaptic models [28, 30]. At presynaptic terminals of glutamatergic synapses, the GABA_B_R can strongly inhibit synaptic activity [31]. Thus, the comodulation of presynaptic behavior by astrocytic glutamate and increasing concentrations of exogenous GABA was considered. Using the model, we can collect neuronal spikes and network data simultaneously and understand the role of astrocytic modulation in response to exogenous GABA by recording the changes in a set of synaptic parameters over time. Numerical simulation shows that the frequency and amplitude of GABA-evoked astrocytic Ca^2+^ oscillations increase with increasing GABA concentrations. Moreover, the enhanced astrocytic glutamate release promotes astrocyte-regulated synaptic release and increases astrocyte-mediated postsynaptic slow inward currents (SICs, i.e., depolarizing currents); both of which can finely tune neuronal excitation. These are efficient and adjustable regulatory mechanisms for balancing the excitation and inhibition of neuronal networks.

## 2. Model and Methods

Based on neurophysiological features and experimental observations, the complete model we developed includes the inhibitory and excitatory neurons, synapses, and astrocytes, as well as the glutamate and exogenous GABA signaling pathways. The response of astrocytes to GABA occurs through activation of GABA_B_Rs. Similar to the activation of astrocytes by glutamate released from presynaptic terminals (red arrows in Figure 1), production of the second messenger inositol 1,4,5-trisphosphate (IP_3_) is triggered, thereby evoking Ca^2+^ oscillations [20]. Ca^2+^ elevation in astrocytes causes glutamate releasing into the extracellular space and ultimately modulating presynaptic vesicle release probability and postsynaptic neuronal excitability (orange arrows). Another important signaling pathway involves the opposing effects of astrocytic glutamate and exogenous GABA at presynaptic terminals of excitatory synapses (blue arrows), where they comodulate synaptic release. Moreover, exogenous GABA can directly regulate the probability of presynaptic GABA release and reshape the activity of postsynaptic GABA_A_Rs [13]. Given that GABA is mainly taken up by the GABAergic neurons [32], the clearance of extracellular GABA by astrocytic uptake is ignored in our model. The model architecture is presented in Figure 1, and subsequent sections describe the mathematical formulas in detail.

### 2.1. Neuron Model

In the present study, the dynamics of a single neuron receiving different stimuli were simulated using a conductance-based leaky integrate-and-fire (LIF) model. This simple spiking model greatly reduces the complexity of neuronal dynamic equation and computational expense, in particular when large groups of the neurons are coupled together into neural astrocytic networks. Both the excitatory and inhibitory neurons are given by different initial values of the model variables. The neuronal model is described by the following equation:

(1) $$\begin{array}{c} \tau_{m}\frac{dv}{dt}=\left(v_{\text{rest}}-v\right)+\left(g_{\text{e}}\left(v_{\text{e}}-v\right)+g_{\text{i}}\left(v_{\text{i}}-v\right)+I_{\text{ex}}\right)\times \frac{1}{g_{\text{leak}}}, \end{array}$$

where *g*_e_, *g*_i_, and *g*_leak_ refer to the total excitatory, inhibitory, and leak conductance, with a reversal potential *v*_e_ = 0 mV and *v*_i_ = −80 mV, respectively. *I*_ex_ is a constant input current, denoting the background current to each neuron. The neuron's membrane potential *v* resets to the default value *v*_rest_ = −60 mV when it reaches the set threshold *v*_th_ = −50 mV. Each spike originating from presynaptic neuron *i* causes a conductance change △*g* in postsynaptic neuron *j*, irrespective of whether the inputs are excitatory or inhibitory [33], i.e., *g*_*j*_ → *g*_*j*_ + △*g*_*ij*_. The postsynaptic conductance can be calculated as follows:

(2) $$\begin{array}{c} \frac{dg_{\text{e}}}{dt}=-\frac{g_{\text{e}}}{\tau_{\text{e}}}, \end{array}$$

(3) $$\begin{array}{c} △g={\bar{g}}_{j}∙r\left(t\right), \end{array}$$

where *τ*_e_ = 5 ms and *τ*_i_ = 10 ms are synaptic time constants, and ${\bar{g}}_{j}$ is the maximal postsynaptic conductance. Excitatory synaptic action was simulated by modeling AMPA and NMDA conductance, while GABA_A_ conductance was modeled to simulate inhibitory synaptic inputs. The item *r*(*t*) is postsynaptic channel open probability, depending on the neurotransmitter concentration in the synaptic cleft (see Equation (22)). The values for neuronal parameters are listed in Table 1.

### 2.2. Astrocyte Model

Unlike the generation of action potentials in the neurons, the computational models describing astrocytic functions always employ astrocytic Ca^2+^ signaling [35]. Following GABA application, GABA_B_R-mediated Ca^2+^ waves depend on the intracellular IP_3_ cascade and are absent in IP_3_R2^−/−^ mice [20]. However, a paucity of exact experimental measurement for GABA-induced IP_3_ activation limits the precise parameters of the IP_3_ dynamic model. Thus, according to experimental results of astrocyte response to GABA [20, 29] and the existing glutamate-activated astrocyte models [24–26], we simplified the model to concentrate only on the IP_3_-evoked Ca^2+^ signaling pathway, in which the rate of IP_3_ production depended on the amount of synaptic glutamate and exogenous GABA in the synaptic cleft. To model the dynamics of Ca^2+^ oscillations, we employed the classical Li–Rinzel model [23]. The modified model of astrocytic IP_3_ production can be explained with the following set of equations:

(4) $$\begin{array}{c} \frac{d\left[{\text{IP}}_{3}\right]}{dt}=\frac{\left({\left[{\text{IP}}_{3}\right]}^{*}-\left[{\text{IP}}_{3}\right]\right)}{\tau_{{\text{IP}}_{3}}}+J_{{\text{GABA}}_{\text{ex}}}+J_{\text{glutamate}}+J_{\text{G}}, \end{array}$$

(5) $$\begin{array}{c} J_{{\text{GABA}}_{\text{ex}}}=\frac{v_{\text{gaba}}^{{\text{IP}}_{3}}∙{\left[{\text{GABA}}_{\text{ex}}\right]}^{n_{1}}}{k_{\text{gaba}}^{n_{1}}+{\left[{\text{GABA}}_{\text{ex}}\right]}^{n_{1}}}, \end{array}$$

(6) $$\begin{array}{c} J_{\text{glutamate}}=\frac{v_{\text{glu}}^{{\text{IP}}_{3}}∙{\left[\text{Glu}\right]}^{n_{2}}}{k_{\text{glu}}^{n_{2}}+{\left[\text{Glu}\right]}^{n_{2}}}, \end{array}$$

where the first equation describes the process of IP_3_ degradation to a steady state at a degradation rate *τ*_IP_3__ = 7 s and an equilibrium concentration [IP_3_]^∗^ = 0.16 *μ*M. The second and third equations describe the production rate of cytoplasmic IP_3_ induced by exogenous GABA and presynaptic glutamate, respectively. [GABA_ex_] and [Glu] are the exogenous GABA and synaptic glutamate concentration, respectively. *v*_gaba_^IP_3_^ and *v*_glu_^IP_3_^ represent the rate of IP_3_ production via GABA and glutamate, respectively, and *k*_gaba_^*n*_1_^ and *k*_glu_^*n*_2_^ are their respective dissociation constants with Hill coefficients *n*_1_ and *n*_2_. Given the amplification interaction between the GABA and glutamate signaling pathways [29], we added a GABA concentration-dependent proportional coefficient *k* to glutamate-induced IP_3_ production:

(7) $$\begin{array}{c} J_{\text{glutamate}}=J_{\text{glutamate}}∙\left(1+k∙\left[{\text{GABA}}_{\text{ex}}\right]\right). \end{array}$$

In our model, the available magnitude of extracellular glutamate and GABA abruptly increases following presynaptic release and exogenous input, respectively, and then exponentially decays. The estimated glutamate (Equation (20)) and GABA concentration in the synaptic cleft can be represented mathematically as follows:

(8) $$\begin{array}{c} \frac{d\left[{\text{GABA}}_{\text{ex}}\right]}{dt}=-g_{\text{GABA}}^{\text{c}}∙\left[{\text{GABA}}_{\text{ex}}\right]∙\Theta \left(t-T_{\text{stim}}\right), \end{array}$$

where *g*_GABA_^c^ is the clearance rate of exogenous GABA with value ln(2)/3 s^−1^ [36]. Θ is the Heaviside function. *T*_stim_ represents the constant stimulus of GABA concentration with a duration 0.5 s [27].

The above dynamic IP_3_ model is similar to the formulation of IP_3_ production in [27]; however, there are some important differences. Firstly, compared with the autoreceptor-mediated astrocyte activation model, the astrocyte model we developed was coactivated by exogenous GABA and synaptically released glutamate. Also, we considered the generation of IP_3_ via gap junction diffusion from neighboring astrocytes in a nonlinear coupling manner [37]. *J*_G_ can be described by the following two equations:

(9) $$\begin{array}{c} J_{\text{G}}=-\frac{F_{\text{ex}}}{2}\left(1+\tanh\left(\frac{{∆}_{ij}{\text{IP}}_{3}-{\text{IP}}_{3}^{\text{thr}}}{\omega }\right)\right)\mathrm{sgn}\left({∆}_{ij}{\text{IP}}_{3}\right), \end{array}$$

(10) $$\begin{array}{c} {∆}_{ij}{\text{IP}}_{3}={\left[{\text{IP}}_{3}\right]}^{i}-{\left[{\text{IP}}_{3}\right]}^{j}, \end{array}$$

where IP_3_^thr^ is the threshold of IP_3_ diffusion at 0.3 *μ*M, *ω* is the scaling factor of diffusion, and *F*_ex_ is the IP_3_ permeability.

Finally, the dynamic equations of astrocytic IP_3_(*t*) are integrated into the Li–Rinzel model to describe the kinetics and properties of Ca^2+^ oscillations in astrocytes:

(11) $$\begin{array}{c} \frac{d\left[{\text{Ca}}^{2+}\right]}{dt}=J_{\text{channel}}-J_{\text{pump}}+J_{\text{leak}}, \end{array}$$

where the three terms denote the calcium flux from the endoplasmic reticulum (ER) to the cytosol gated by IP_3_ (*J*_channel_), the leakage flux from the ER (*J*_leak_), and Ca^2+^ reuptake from the cytosol to the ER via ATP-dependent pumps (*J*_pump_), respectively. For the sake of simplicity, the expansion of terms is omitted and the three fluxes and parameters refer to those in [38].

When IP_3_-induced elevation in Ca^2+^ concentration exceeds the threshold *C*_*θ*_ at time *t*_*j*_, a fraction *r*_A_(*t*_*j*_) of astrocytic glutamate resources can be released into the extracellular space by vesicle exocytosis [39]. The fraction of readily releasable is given as follows:

(12) $$\begin{array}{c} r_{\text{A}}\left(t\right)=U_{\text{A}}∙x_{\text{A}}\left(t\right), \end{array}$$

where *U*_A_ is the resting glutamate release probability and *x*_A_ is the fraction of available glutamate resources for release, according to the following:

(13) $$\begin{array}{c} \frac{dx_{\text{A}}}{dt}=\frac{1-x_{\text{A}}}{\tau_{\text{G}}}-r_{\text{A}}\left(t\right)∙\delta \left(t-t_{j}\right), \end{array}$$

where *τ*_G_ is the glutamate resource reintegration time constant. The astrocyte-derived glutamate concentration *G*_A_ in the extrasynaptic cleft is described as follows:

(14) $$\begin{array}{c} \frac{dG_{\text{A}}}{dt}=-g_{\text{A}}^{\text{c}}∙G_{\text{A}}+r_{\text{A}}∙\varrho_{\text{e}}∙G_{\text{T}}∙\delta \left(t-t_{j}\right)∙\left(1+k∙\left[{\text{GABA}}_{\text{ex}}\right]\right), \end{array}$$

where *g*_A_^c^ is the clearance rate of glutamate, *ϱ*_e_ denotes the volume ratio of vesicles to periastrocytic space, and *G*_T_ is the total vesicular glutamate concentration in astrocytes. The parameters are given in Table 2.

### 2.3. Synapse Model

The effects of astrocytic glutamate and exogenous GABA on presynaptic terminals are mediated by activation of mGluRs and GABA_B_Rs, respectively. Both of these receptor types regulate the amount of Ca^2+^ influx into presynaptic terminals; the former promotes [40] and the latter retards [41]. Release of vesicles is dependent on elevation in intracellular Ca^2+^ concentration [42]. Therefore, open proportion *U* of Ca^2+^ channels modulated by the two transmitters is a critical parameter that decides the probability of presynaptic neurotransmitter release. To mimic the effects of astrocytic glutamate and exogenous GABA comodulation on synaptic release probability, we used a modified kinetic model of synaptic release regulated by astrocyte [28], which is based on the Tsodyks–Markram (TM) phenomenological model of synaptic activity [43], and added GABA activation kinetic scheme. The corresponding kinetic equation reads as follows:

(15) $$\begin{array}{c} U=U_{0}+\left(\xi -U_{0}\right)∙\Gamma -U_{0}∙r_{{\text{GABA}}_{\text{B}}}, \end{array}$$

where *U*_0_ is defined as a constant in the TM model [44], denoting the open ratio of Ca^2+^ channels induced by action potentials, i.e., resting synaptic release probability. The second term is the effect of astrocyte-released glutamate on presynaptic glutamate receptors, in which Γ is the proportion of activated receptors and parameter *ξ* (0 ≤ *ξ* ≤ 1) determines the type and strength of the action of astrocytes on presynaptic terminals. The third term denotes the probability of modulation of synaptic basal release by GABA, and *r*_GABA_B__ is the fraction of GABA_B_-mediated Ca^2+^ channels that close. The probability that channels are open or closed is determined by the following:

(16) $$\begin{array}{c} \frac{d\Gamma }{dt}=O_{\text{G}}∙G_{\text{A}}∙\left(1-\Gamma \right)-\Omega_{\text{G}}∙\Gamma , \end{array}$$

(17) $$\begin{array}{c} \frac{dr_{{\text{GABA}}_{\text{B}}}}{dt}=\alpha_{{\text{GABA}}_{\text{B}}}∙\left[{\text{GABA}}_{\text{ex}}\right]∙\left(1-r_{{\text{GABA}}_{\text{B}}}\right)-\beta_{{\text{GABA}}_{\text{B}}}∙r_{{\text{GABA}}_{\text{B}}}, \end{array}$$

where [GABA_ex_] and *G*_A_ represent the concentrations of exogenous GABA and astrocyte-released glutamate, respectively, given by Equation (8) and Equation (14). The parameters *O*_G_ and *Ω*_G_ are the forward and backward rate constants for astrocytic glutamate binding to excitatory presynaptic receptors, respectively, and *α*_GABA_B__ and *β*_GABA_B__ are the rate constants of GABA_B_R-mediated binding or unbinding, respectively.

Accordingly, the modified resting synaptic release probability *U* will determine the fraction *u*_S_ of available neurotransmitter to be utilized occurring at each presynaptic spike time *t*_*k*_:

(18) $$\begin{array}{c} \frac{du_{\text{S}}}{dt}=\frac{-u_{\text{S}}}{\tau_{\text{fac}}}+U∙\left(1-u_{\text{S}}\right)∙\delta \left(t-t_{k}\right), \end{array}$$

where *τ*_fac_ is the relaxation time constant of facilitation and determines the rate of *u*_S_ decaying to zero in the absence of spikes. The fraction of total neurotransmitter available for release *x*_S_ is described by the following:

(19) $$\begin{array}{c} \frac{dx_{\text{S}}}{dt}=\frac{1-x_{\text{S}}}{\tau_{\text{rec}}}-r_{\text{S}}∙\delta \left(t-t_{k}\right), \end{array}$$

where *τ*_rec_ is the recovery time constant and determines the reintegration rate of resources to the available pool. *r*_S_ denotes the fraction of neurotransmitter effectively released into the extracellular space, i.e., probability of neurotransmitter release (Pr), defined as *r*_S_ = *u*_S_∙*x*_S_. The estimated glutamate concentration *G*_S_ from presynaptic release can be represented mathematically as follows:

(20) $$\begin{array}{c} \frac{dG_{\text{S}}}{dt}=-g_{\text{S}}^{\text{c}}∙G_{\text{S}}+r_{\text{S}}∙\varrho_{\text{c}}∙Y_{\text{T}}∙\delta \left(t-t_{k}\right), \end{array}$$

where *g*_S_^c^ is the clearance rate of glutamate via neuronal and astrocytic uptake or spillover (flowing out of the synaptic cleft). *ϱ*_c_ is the vesicular to mixing volume ratio, and *Y*_T_ represents the total vesicular glutamate concentration in the presynaptic bouton. Akin to those described in glutamate release process in Equations (18)–(20), when a single action potential arrived at GABAergic synapse, GABA in synaptic vesicles are released from presynaptic terminal and then diffuse in the synaptic cleft, where they are retrieved by endocytosis [45]. Because this study focused on the regulation of astrocytes on the excitatory neurons, the open proportion *U* in presynaptic terminal of GABAergic synapse was set a constant for simplification.

Once vesicles are released from presynaptic terminals or astrocytes, glutamate diffuses across the synaptic cleft and binds to postsynaptic AMPA and NMDA receptors, resulting in an increase in conductance. The dynamics of the synaptic conductance gating variable *r*(*t*) in Equation (3) can be represented using a two-state model [46]. Transition between closed and open states of the channel is considered a Markov process based on the following diagram:

(21) $$\begin{array}{c} C+T\begin{array}{c} \alpha \\ ⇌\\ \beta \end{array}O, \end{array}$$

where *C* and *O* indicate the unbound and bound states of the channel to neurotransmitter, respectively, *T* is the glutamate or GABA concentration, and *α* and *β* are the forward and backward rate constants, respectively. The two-state kinetic model describes the process of direct receptor binding to neurotransmitter, changing the ion channel. The fraction of the receptors in the open state *r* is described by the first-order dynamic equation:

(22) $$\begin{array}{c} \frac{dr}{dt}=\alpha ∙\left[T\right]∙\left(1-r\right)-\beta ∙r. \end{array}$$

Finally, NMDA-, AMPA-, and GABA_A_-mediated postsynaptic currents are expressed as functions of *r*(*t*) and the membrane potential *v* by the following equations [46]:

(23) $$\begin{array}{c} I_{\text{AMPA}}={\overset{¯}{g}}_{\text{AMPA}}∙r\left(t\right)∙\left(v-E_{\text{AMPA}}\right), \end{array}$$

(24) $$\begin{array}{c} I_{\text{NMDA}}={\overset{¯}{g}}_{\text{NMDA}}∙\text{Mg}\left(v\right)∙r\left(t\right)∙\left(v-E_{\text{NMDA}}\right), \end{array}$$

(25) $$\begin{array}{c} I_{{\text{GABA}}_{\text{a}}}={\overset{¯}{g}}_{{\text{GABA}}_{\text{A}}}∙r\left(t\right)∙\left(v-E_{{\text{GABA}}_{\text{A}}}\right), \end{array}$$

where $\overset{¯}{g}$ is the maximum conductance, $\;{\overset{¯}{g}}_{\text{AMPA}}=0.35$ nS, ${\overset{¯}{g}}_{\text{NMDA}}=0.1$ nS, ${\overset{¯}{g}}_{{\text{GABA}}_{\text{A}}}=0.62$ nS, *v* is the postsynaptic membrane potential, *E* is the synaptic reversal potential, *E*_AMPA_ = *E*_NMDA_ = 0 mV, and *E*_GABA_A__ = −80 mV. Notably, a unique property of NMDA currents is that NMDA receptors contain a voltage-dependent term representing magnesium (Mg^2+^) block at [Mg^2+^] = 1 mM [47]:

(26) $$\begin{array}{c} \text{Mg}\left(v\right)=\frac{1}{1+\exp\left(-0.062*v\right)\left[{\text{Mg}}^{2+}\right]/3.57}. \end{array}$$

The slow inward current *I*_sic_ elicited by astrocytic glutamate can be defined as follows [48, 49]:

(27) $$\begin{array}{c} I_{\text{sic}}\left(t\right)=I_{\text{NMDA}}\left(t\right)+I_{\text{AMPA}}\left(t\right). \end{array}$$

In this fashion, postsynaptic mechanisms of astrocytic glutamate regulation mediated by NMDA and AMPA receptors complicate the characterization of regular postsynaptic currents by glutamate released from presynaptic terminals. Thus, the two types of excitatory events (SICs and EPSCs) can be distinguished according to their origin, astrocyte-derived glutamate *G*_A_ (Equation (14)) and synaptically released glutamate *G*_S_ (Equation (20)), respectively. Noted worthily, although the NMDA receptors that mediate SICs and EPSCs are different [50], NMDA receptor subtypes are often not distinguished in the computational models for simplicity. The parameters for the synapse model are listed in Table 3.

### 2.4. Neuronal–Astrocyte Network

Based on the network components mentioned above, we simulated a two-dimensional network model (Figure 2). Each neuron and astrocyte were assigned a spatial location in a square grid with dimensions of 10 × 10 mm planar units, providing a suitable physical arrangement for signaling transmission among them [51]. The neuronal network model comprises 400 excitatory and 100 inhibitory neurons with 0.2 connection probability as well as 400 astrocytes. Experimental results show that individual cortical astrocyte can enwrap the nearby neurons within its territory and modulate the synapses associated with hundreds of dendrites [52]. According to their spatial coordinates, therefore, we calculated the minimum distance between astrocytes and the pre- and postsynaptic neurons and then determined which astrocyte should be responsible for this synapse. Connection between astrocytes was also based on their coordinates. Considering a mean numerical density of astrocytes of 17,575 cells per mm^3^ in the rat visual cortex [53], average intersomal distance between astrocytes was set 675 *μ*m in our model by enlarging in proportion. In this way, an astrocyte can be connected to about 100 nearby excitatory synapses and 4 astrocytes on average. Multiple variables were calculated and recorded during each 10 s simulation, including neuronal firing, astrocytic calcium oscillations, and excitatory presynaptic release. The model was implemented in the Brian 2.0 simulator [54, 55].

## 3. Results

### 3.1. Astrocytic Glutamate Increases the Average Network Firing Rate

We began our analysis by describing the firing behavior of the neurons. The neural-astrocytic network was treated with increasing GABA concentrations (0, 1, 5, and 10 *μ*M). A quarter of the neurons were chosen for clarification using raster plot (Figure 3). The network firing rate, measured as an average across the spikes of all neurons (time bin width *∆t* = 1 ms), is shown in the bottom panel of the raster plot of neuronal firing. Furthermore, we fixed inhibitory synaptic release probability at a constant of 0.5 [56] to ignore the effect of GABA_B_R-mediated disinhibition at inhibitory presynaptic terminals. In order to produce weak and strong inhibitory effects on excitatory inputs, maximal conductance of GABA_A_ increases with the change of exogenous concentration depending on the experimental results [13]. Figures 3(a)–3(d) (top panel) show that the firing activity of the excitatory (red) and inhibitory (blue) neurons during treatment with different concentrations of GABA decreased, in line with the previous experimental observation that we performed acute GABA treatment on the cortical cultures [57]. The release time of gliotransmitter glutamate (green) from astrocytes was significantly affected. Astrocytic glutamate triggered synchronized responses in the neurons, which increased the average network firing rate (bottom panel). The synchronized neuronal activities are consistent with the results of electrophysiological experiments [50, 58] and computational simulation [59], which imply that astrocytes have a vital role in modulation the firing of the neurons.

### 3.2. GABA-Activated Astrocytes Augment Calcium Oscillations and Glutamate Release

The key model parameters for GABA-induced astrocytic activity are shown in Figure 4, including the intracellular cascade of IP_3_-mediated Ca^2+^ response and Ca^2+^-dependent glutamate release. The dynamic changes in intracellular Ca^2+^ in astrocyte were regulated by the integration of the exogenous GABA and presynaptic glutamate signaling pathways (Figure 1), akin to spatial and temporal integrators [60]. With the exogenous GABA concentration increased ([GABA_ex_] = 0, 1, 5, and 10 *μ*M), the concentration of glutamate resulting from presynaptic release decreased significantly (Figure 4(a)), while the activation of glutamate receptors on astrocyte increased (Figure 4(b)). This may be attributed to the amplification of mGluRs via crosstalk with the GABA_B_Rs [29]. In these cases, compared to the condition without exogenous stimuli (Figure 4(c), black line), the time course of IP_3_ production differed across the three paradigms due to the increase of GABA concentrations ([GABA_ex_] = 1, 5, and 10 *μ*M) in the synaptic cleft (Figure 4(c), colored lines), which resulted in greater Ca^2+^ oscillatory behavior (Figure 4(d)). In the Ca^2+^ variation curve, the single pulse elevation may arise from direct stimulation with exogenous GABA, and the subsequent long-lasting Ca^2+^ oscillations could be evoked by glutamate [27]. Indeed, the astrocytic Ca^2+^ response closely depends on the amount of glutamate released from presynaptic terminals in the synaptic cleft [51]. Although the neurons were suppressed, an amplification interaction between the GABA and glutamate signaling pathways augmented the amplitude and frequency of Ca^2+^ oscillations in astrocyte. Simulated results indicate that a higher concentration of GABA leads to a stronger and prolonged Ca^2+^ wave, which changes the rate of glutamate release (Figure 4(e)). Nevertheless, there are no experimental data available to precisely quantitate the effect of these two receptors. Further experimental studies are required to elucidate the exact mechanism and quantitative properties of Ca^2+^ oscillations evoked by multiple neurotransmitters.

### 3.3. Enhanced Astrocytic Glutamate Promotes Presynaptic Release

The variations in presynaptic release probability in our model were regulated by astrocytic glutamate and exogenous GABA (Figure 1). As a contrast, the direct response of presynaptic terminal to exogenous GABA in the absence of astrocytic modulation is shown in Figure 5(a). The release probability Pr significantly decreased with GABA inhibition, while Pr in central excitatory synapses was between 0.1 and 0.9 [61]. This indicates that increased GABA concentrations robustly inhibit excitatory presynaptic release [31]. In the presence of astrocyte-derived glutamate, the scenario could be reversed (Figure 5(b)). In particular, the regulation of presynaptic release by astrocyte-derived glutamate was significantly enhanced as the concentration of exogenous GABA increased. The rate of astrocytic glutamate potentiation was larger than the rate of GABA depression, which gave rise to an increase in Pr, illustrating that glutamate exocytosis from astrocytes promoted presynaptic transmitter release [40]. Furthermore, the variations in excitatory postsynaptic currents (EPSCs) elicited by presynaptic glutamate release are consistent with the quantal size variability in presynaptic vesicle release (Figure 6). The results suggest that exogenous GABA causes a large decrease in the EPSC amplitude [14], whereas the release of astrocytic glutamate enhances excitatory postsynaptic currents.

### 3.4. Astrocyte-Mediated Slow Inward Currents Increase Postsynaptic Neuronal Excitability

Both excitatory and inhibitory inputs to the postsynaptic neurons are accompanied by a decrease in impedance and an increase in membrane conductance [33]. The inhibitory and excitatory synaptic conductance values *g*_i_ and *g*_e_ were consistently balanced at a certain ratio [62]; the former was several fold higher than the latter [63]. In our model, postsynaptic events were characterized by changes in current instead of changes in conductance. To investigate the impact of NMDAR- and AMPAR-mediated SICs on the postsynaptic neurons, we removed the excitatory effect of regular synaptic currents driven by synaptically released glutamate. These results could be the direct response of the postsynaptic neuron to astrocyte.

GABA-evoked astrocytic Ca^2+^ oscillations triggered the release of glutamate (Figure 7(a)), which diffused into the extracellular space and bound to post-extrasynaptic glutamate receptors, eliciting depolarizing SICs (Figures 7(b)–7(e)). Astrocyte-mediated SICs caused membrane depolarization in the postsynaptic neurons, which was sufficient to reach the firing threshold and ultimately influenced the time course of postsynaptic neuronal firing (Figure 7). Pathological conditions, such as neuronal depolarization, termed paroxysmal depolarization shifts, may contribute to seizure generation [64]. Indeed, intracellular Ca^2+^ elevation in astrocytes is a crucial factor in the regulation of SICs, which has been previously reported in *in vitro* [49] and numerical studies [48, 65]. Moreover, the SIC amplitude is determined by the extracellular glutamate concentration. Both an enhanced astrocytic glutamate release and a downregulated glutamate clearance rate can dramatically modulate neuronal excitability, therefore increasing seizure susceptibility [48, 66, 67]. The results of this simulation show that the higher concentration of exogenous GABA is injected to neuronal-astrocytic network, the larger amplitude of astrocyte-mediated SICs is evoked due to the enhanced release of astrocytic glutamate. The increase in excitability could partly counteract the resulting decrease in EPSCs induced by presynaptic glutamate, thereby fine-tuning neuronal network excitation.

## 4. Discussion and Conclusions

Numerous *in vitro* and *in vivo* studies indicate that astrocytes play a vital role in neuronal excitability and synaptic transmission. Based on neurophysiological findings [20], we developed a biophysical neuronal-astrocytic network model to quantitatively analyze the impact of astrocytes on the modulation of neuronal excitability at different concentrations of exogenous GABA. This is an important issue in view of recent studies regarding the mechanism of the GABAergic neuron to astrocyte signaling, and the simulation results give important clues to the involved GABA signaling mechanism.

Our research yielded several predictions. Firstly, the period and amplitude of Ca^2+^ signaling were dramatically elevated by increasing GABA dose strength. Without exogenous stimulus, i.e., [GABA_ex_] = 0 *μ*M, neuronal activity can also trigger relatively slower astrocytic Ca^2+^ oscillations. In fact, astrocyte Ca^2+^ events occur in a slow and prolonged manner under physiological condition [68]. This is probably due to the full intracellular cascade of glutamate-activated astrocyte requiring successive events including astrocytic mGluR activation, second messenger IP_3_ production, astrocyte Ca^2+^ elevation, and astrocytic gliotransmitter release. Consistent with [20], our results show that exogenous GABA produces a concentration-dependent increase in the elevation rate of astrocyte Ca^2+^.

It is known that astrocytes release glutamate through multiple pathways [69], in which Ca^2+^-dependent exocytosis may be the most widely examined. Considering the spontaneous astrocytic Ca^2+^ oscillations [70], neuronal activity, or external stimulus-induced Ca^2+^ increase [71], there seems to be a consensus that increased Ca^2+^ concentration results in glutamate release and subsequent neuronal regulation. Yet, Ca^2+^-dependent mechanism remains a controversial topic. Recent study suggests that Ca^2+^-dependent gliotransmission is a pharmacological phenomenon rather than a physiological process [72]. Given the complexity of astrocyte Ca^2+^ activity [73], it is not surprising that the literatures report some discrepant results regarding the mechanisms of glutamate release and gliotransmission. Although the mechanism is not fully settled, a number of published astrocyte computational models have been based on astrocytic Ca^2+^ signaling [35]. Our model also considers Ca^2+^-dependent mechanism as the method of glutamate release from astrocytes. Numerical results in this paper verify astrocyte function as the conversion of GABA inhibition into glutamatergic excitation, in which astrocytic Ca^2+^ activity is a crucial factor contributing to network excitability. Although the release of synaptic glutamate was inhibited by GABA, astrocyte Ca^2+^ response in this model was enhanced, which may be the amplifying interaction between the GABA_B_R and mGluR-induced Ca^2+^ signaling [29]. If these are further verified by experimentation, irrespective of which neurotransmitter excites astrocytes, an intervention in Ca^2+^ signaling may be a potential mechanism for some drug targets. For instance, anticonvulsants reduce neuronal excitability by blocking astrocytic Ca^2+^ signaling [64].

Another significant finding of our model is that GABA and astrocytic glutamate play opposing roles at excitatory presynaptic terminals. We used neurotransmitter depletion and reintegration to describe the modulation of basal release probability by these two factors. The net effect of GABA and astrocytic glutamate on excitatory presynaptic terminals is due to the coexistence of mixed scenarios. The results suggest that the enhanced release of astrocytic glutamate results in stronger vesicle recruitment and release as compared with the inhibitory effect of GABA. From the perspective of information transmission, the probability of presynaptic glutamate release depends on the pattern of presynaptic activity that integrates the contradictory effects of GABA and astrocytic glutamate. Thus, the synapse can be thought of as a filter [74], determining whether synaptic information is transmitted to the postsynaptic neurons.

Our model illustrates that astrocyte-elicited SIC by activation of extrasynaptically located postsynaptic NMDA receptors is the other mechanism that affects neuronal activity. Unlike the results of postsynaptic high frequency activity produced by SICs in pathological conditions [48, 66, 75], SIC-mediated increase of neuronal excitability in our study seems to be slightly in modulation of amplitude and period. This scenario may result from integrated inhibitory inputs to the postsynaptic neurons, which are connected to about 20 inhibitory neurons in our model. In fact, SICs can be amplified by upregulating mGluRs on astrocytes, but this was commonly observed in pathological tissues such as epilepsy [76]. Although it is hard to fight against the extra amount of GABA, these results evidence the involvement of astrocytes in modulation of neuronal activity, suggesting that astrocytic glutamate mediates the increase of excitation in the neural-astrocyte network.

Overall, the model described in the present study attempts to mimic the bidirectional neuron-astrocyte interaction under exogenous stimuli. These results demonstrate the involvement of astrocytes in synaptic transmission and suggest the excitatory drive of GABA-activated astrocytes in the neuronal network. Indeed, there exists a fine balance between excitation and inhibition in the central nervous system. Astrocytes have the potential ability to modulate synaptic activity and maintain this excitatory-inhibitory balance in particular brain states, which is far-reaching within brain function.

## Figures and Tables

**Figure 1:** The main pathways of exogenous GABA (GABA_ex_) action in the tripartite glutamatergic synapse model. Red arrows indicate the glutamatergic gliotransmission pathways, including astrocytic metabotropic glutamate receptor (mGluR) activation, IP_3_-gated Ca^2+^ mobilization, astrocytic glutamate release, presynaptic mGluR activation, and postsynaptic AMPAR and NMDAR-mediated depolarization currents. The orange and blue arrows represent the regulation of the astrocyte and presynaptic neuron by exogenous GABA, respectively. GABA_ex_ represents simulated GABA injection to the neuronal-astrocytic model. ER refers to the endoplasmic reticulum. It is necessary to note that locations of astrocytic and neuronal receptors in this figure do not represent their exact physiological distribution.

**Figure 2:** The 2D neural astrocytic network model. Astrocytes, the inhibitory neurons, and the excitatory neurons are represented by green stars and blue and red dots, respectively. Green lines represent astrocyte network and the neuronal connections are omitted for clarity.

**Figure 3:** The raster plot and mean firing rate of neural activity during treatment with different concentrations of GABA: (a) 0 *μ*M, (b) 1 *μ*M, (c) 5 *μ*M, and (d) 10 *μ*M. The top panel shows astrocytic glutamate release (green) and excitatory (red) and inhibitory (blue) neuronal firing. The average network firing rate is shown at the bottom.

**Figure 4:** The dynamic response of astrocyte to presynaptic glutamate and exogenous GABA. (a) The amount of presynaptically released glutamate (Glu_syn_) decreases as the concentration of exogenous GABA increases, but (b) there is greater activation of mGluRs on astrocyte due to the crosstalk with GABA_B_ receptors, which results in (c) IP_3_ production and (d) IP_3_-gated [Ca^2+^] elevation. (e) Once the [Ca^2+^] threshold has been reached (0.2 *μ*M, red dashed line), astrocyte releases glutamate (Glu_astro_) into the extracellular space. To avoid triggering repeatedly the release in all the time steps, gliotransmitter release event is triggered only once in threshold conditions, a mechanism similar to the refractory period of the neuron.

**Figure 5:** Variations in presynaptic glutamate release probability (Pr) during (a) astrocyte-independent and (b) astrocyte-dependent pathways. The dots represent each presynaptic release event.

**Figure 6:** Variations in excitatory postsynaptic currents (EPSCs) induced by glutamate released from presynaptic terminal during treatment with different concentrations of GABA: (a) 0 *μ*M, (b) 1 *μ*M, (c) 5 *μ*M, and (d) 10 *μ*M.

**Figure 7:** Astrocyte-mediated SICs and the change in postsynaptic membrane potential. (a) Enhanced glutamate release by astrocytes due to the elevated concentrations of GABA ((b–e) [GABA_ex_] = 0 *μ*M, 1 *μ*M, 5 *μ*M, and 10 *μ*M) results in a stronger *I*_sic_ and subsequently makes the neurons more excitable to resist the increased GABA inhibition.

**Table 1:** Parameters used in the neuronal model [34].

Parameter	Description	Value
*τ*_m_	Membrane time constant	20 ms
*v*_th_	Firing threshold	-50 mV
*v*_rest_	Resting potential	-60 mV
*v*_e_	Excitatory reversal potential	0 mV
*v*_i_	Inhibitory reversal potential	-80 mV
*g*_leak_	Leak conductance	10 nS
*I*_ex_	Background current	105 pA
*τ*_ref_	Absolute refractory period	5 ms
*τ*_e_	Excitatory conductance decay time constant	5 ms
*τ*_i_	Inhibitory conductance decay time constant	10 ms

**Table 2:** Parameters used in the astrocyte model [24, 28, 37].

Parameter	Description	Value
IP_3_^∗^	Steady-state concentration of IP_3_	0.16 *μ*M
*τ*_IP_3__	IP_3_ degradation constant	7 s
*v*_gaba_^IP_3_^	Rate of IP_3_ production via GABA	0.1625 *μ*M s^−1^
*v*_glu_^IP_3_^	Rate of IP_3_ production via glutamate	0.062 *μ*M s^−1^
*n*_1_	GABA Hill coefficient	0.3
*n*_2_	Glutamate Hill coefficient	0.2
*k*_GABA_^*n*^	Dissociation constant for GABA-stimulated IP_3_ production	0.6 *μ*M
*k*_glu_^*n*^	Dissociation constant for glutamate-stimulated IP_3_ production	0.78 *μ*M
IP_3_^thr^	Threshold for IP_3_ diffusion	0.3 *μ*M
*F*_ex_	IP_3_ permeability	0.09 *μ*M s^−1^
*ω*	Scaling factor of IP_3_ diffusion	0.05 *μ*M
*C*_*θ*_	Ca^2+^ threshold for exocytosis	0.2 *μ*M
*τ*_G_	Glutamate reintegration time constant	1.66 s
*U*_A_	Resting glutamate release probability	0.6
*ϱ*_e_	Volume ratio of vesicles to periastrocytic space	6.5 × 10^−4^
*g*_A_^c^	Clearance rate of astrocytic glutamate	60 s^−1^
*G*_T_	Total vesicular glutamate concentration	200 mM
*k*	GABA concentration-dependent proportionality coefficient	0.3

**Table 3:** Parameters used in the synapse model [28, 46].

Parameter	Description	Value
*U*_0_	Resting synaptic release probability	0.3
*ξ*	Type and strength of astrocytes acting on presynapses	0.8
*O*_G_	Activation rate of astrocytic glutamate	1.5 M^−1^ s^−1^
*Ω*_G_	Inactivation rate of astrocytic glutamate	0.2 s^−1^
*α*_GABA_B__	GABA_B_ forward rate constant	16 *μ*M^−1^ s^−1^
*β*_GABA_B__	GABA_B_ backward rate constant	6 s^−1^
*τ*_fac_	Facilitation time constant	0.3 s
*τ*_rec_	Recovery time constant	0.5 s
*g*_S_^c^	Presynaptic glutamate clearance rate	40 s^−1^
*ϱ*_c_	Vesicular to mixed volume ratio	0.005
*Y*_T_	Total vesicular glutamate concentration	500 mM
*α*_AMPA_	AMPA forward rate constant	1.1 *μ*M^−1^ s^−1^
*β*_AMPA_	AMPA backward rate constant	190 s^−1^
*α*_NMDA_	NMDA forward rate constant	0.072 *μ*M^−1^ s^−1^
*β*_NMDA_	NMDA backward rate constant	6.6 s^−1^
*α*_GABA_A__	GABA_A_ forward rate constant	0.53 *μ*M^−1^ s^−1^
*β*_GABA_A__	GABA_A_ backward rate constant	180 s^−1^
*g*_GABA_^uptake^	GABA reuptake rate constant	6 s^−1^

## Data Availability

The data in this study are available on request from the corresponding author. The data are not publicly available due to privacy or ethical restrictions.
